The article "Species-specific chemosensory gene expression in the olfactory organs of the malaria vector Anopheles gambiae" was retracted in 2015. Reasons: contaminated cell lines or tissues; errors in the data; unreliable results or conclusions.

# Species-specific chemosensory gene expression in the olfactory organs of the malaria vector *Anopheles gambiae*

**DOI:** 10.1186/1471-2164-15-1089

**Published:** 2014-12-11

**Authors:** Theresa K Hodges, Luciano V Cosme, Giridhar Athrey, Sharmila Pathikonda, Willem Takken, Michel A Slotman

**Affiliations:** Department of Entomology, Texas A&M University, College Station, TX 77843 USA; Laboratory of Entomology, Wageningen University, Wageningen, The Netherlands

## Abstract

**Background:**

The malaria mosquito *Anopheles gambiae* has a high preference for human hosts, a characteristic that contributes greatly to its capacity for transmitting human malaria. A sibling species, *An. quadriannulatus,* has a quite different host preference and feeds mostly on bovids. For this reason it does not contribute to human malaria transmission. Host seeking in mosquitoes is modulated by the olfactory system, which is primarily housed in the antennae and maxillary palps. Therefore, the detection of differing host odors by sibling species may be reflected in the expression level of the olfactory genes involved. Accordingly, we compared the transcriptomes of the antennae and maxillary palps of *An. gambiae* and *An. quadriannulatus.*

**Results:**

We identified seven relatively abundant olfactory receptors, nine ionotropic receptors and three odorant binding proteins that are substantially up-regulated in *An. gambiae* antennae. Interestingly, we find that the maxillary palps of *An. gambiae* contain a species-specific olfactory receptor*, Or52,* and five *An. gambiae-*specific gustatory receptors (*AgGr48-52*) that are relatively abundant. These five gustatory receptors are also expressed in *An. gambiae* antennae, although at lower level, indicating a likely role in olfaction, rather than gustation. We also document an approximately three-fold higher overall expression of olfaction genes in the maxillary palps of *An. quadriannulatus,* indicating an important role of this organ in the olfaction system of this species. Finally, the expression of the CO_2_ receptor genes is five to six-fold higher in the zoophilic *An. quadriannulatus,* implying a much higher sensitivity for detecting CO_2_*.*

**Conclusions:**

These results identify potential human host preference genes in the malaria vector *An. gambiae.* Interestingly, species-specific expression of several gustatory receptors in the olfactory organs indicate a role in olfaction rather than gustation. Additionally, a more expansive role for maxillary palps in olfaction is implicated than previously thought, albeit more so in the zoophilic *An. quadriannulatus.*

**Electronic supplementary material:**

The online version of this article (doi:10.1186/1471-2164-15-1089) contains supplementary material, which is available to authorized users.

The article "Species-specific chemosensory gene expression in the olfactory organs of the malaria vector Anopheles gambiae" was retracted in 2015. Reasons: contaminated cell lines or tissues; errors in the data; unreliable results or conclusions.

## Background

The malaria mosquitoes within the *Anopheles gambiae* complex vary considerably in their host preference. Africa’s main malaria vector *An. gambiae s.s.* is highly anthropophilic, whereas the zoophilic *An. quadriannulatus* rarely if ever attacks humans [1]. This preference of *An. gambiae* for human hosts is a major factor in its high vectorial capacity for human malaria parasites. Conversely, although the zoophilic *An. quadriannulatus* is a competent malaria vector [2], this species does not contribute to malaria transmission because it rarely feeds on human hosts in the field, although it does so readily in the lab [3, 4].

Mosquitoes’ host attraction is primarily modulated by the olfaction system and *An. gambiae* females are strongly attracted to emanations from human sweat. Volatiles produced by microflora on the surface of human skin are believed to be responsible for the uniqueness of human odor [5, 6]. Over 350 volatiles are found in human sweat [7], and while not all of these play a role in allowing *An. gambiae* to differentiate human hosts from others, it is likely that a blend of human volatiles is involved. For example, *An. gambiae* females are attracted to a mixture of ammonia, lactic acid, as well as a synergistic blend of ammonia, lactic acid and carboxylic acids [8–10]. *Anopheles gambiae* and *An. quadriannulatus* also show different sensitivities to various compounds found in human and animal sweat and/or breath. Therefore, the relative quantities of the constituents of host odor blends, rather than the presence or absence of specific volatiles, could be important in determining attractiveness to various species [11, 12].

The antennae and the maxillary palps, the two main olfactory appendages of *An. gambiae* [13, 14], are lined with sensilla that house the olfactory sensory neurons that express olfactory receptors (ORs) [15] or ionotropic receptors (IRs) [16, 17]. The binding of odorants to the ORs and IRs triggers the transduction cascade that sends a signal to the olfactory lobes in the cerebral ganglion of the insects [18]. Because of this direct interaction between the receptors and the odorants, differences in host preference between species may be reflected in differences in the expression or molecular structure of the receptors.

Currently, 76 *Ors* ([19, 20] and 44 *Irs* have been identified [21]). ORs are heteromeric ligand-gated ion channels encoded by the highly conserved co-receptor *Orco* and a specific *Or*. ORs differ in their tuning breadth and some ORs respond to either a single or small number of odorants, while others respond to a variety of volatiles [22–26]. IRs are also heteromeric ligand-gated ion channels, but these can contain up to three different subunits that include one or two of the broadly expressed co-receptors *Ir25a* and *Ir8a* [16, 26].

The article "Species-specific chemosensory gene expression in the olfactory organs of the malaria vector Anopheles gambiae" was retracted in 2015. Reasons: contaminated cell lines or tissues; errors in the data; unreliable results or conclusions.

In addition to the ORs and IRs, odorant binding proteins (OBPs) play a role in odorant recognition and interact directly with odorants. OBPs are small, water-soluble transport molecules abundant in the lymph of the sensilla. They transport hydrophobic odorants through the haemolymph to the receptors (reviewed in [27]). Currently, 57 putative *Obp*s have been identified [28–30], but only 34 *Obps* are expressed in female antennae [31]. Some OBPs almost certainly play a role in the transport of molecules outside the olfaction system, as two *Obps* are known to be expressed only in female heads [17].

Differences in the expression level of olfaction genes have been observed between closely related species feeding on different hosts. Expression levels of as many as 53% of the ORs and 55% of the OBPs in the antennae differed between the generalists *D. melanogaster, D. simulans*, and their specialist sister-species *D. sechellia* which feeds on the toxic *Morinda citrifolia* pairs. This is a significantly higher number than observed in other genes [32]. Although some of these changes may be due to neutral evolution, several genes have undergone a major change in expression level along the *D. sechellia* branch, and are thought to be associated with host shifts [32]. For example, Or22a is strongly up-regulated in *D. sechellia.* This receptor is sensitive to a compound emitted by the fruit of *D. sechellia’*s host plant *Morinda citrifolia* [33]. Additionally, *D. sechellia* lost six *Or* genes since its split from its generalist sister-species *D. simulans,* which lost none [34]. Furthermore, an increase in olfactory receptor loss was also associated with host specialization in *D. erecta* [35] *.* Recently, a comparison between the day-time transcriptome of *An. gambiae* and *An. quadriannulatus* antennae identified differences in olfaction gene expression that may be related to the difference in host preference between these sibling species [36]. It has been shown however that olfactory gene expression fluctuates across the circadian cycle [37]. Here, we compare the transcriptome of both the female antennae and palps of the anthropophilic *An. gambiae* and the zoophilic *An. quadriannulatus,* during the early dark cycle, when both species are actively seeking hosts [38, 39]. These comparisons further show the divergence of the olfactory organs of these two species, and allows us to identify species-specific chemosensory genes in *An. gambiae* that may be responsible for human host preference.

The article "Species-specific chemosensory gene expression in the olfactory organs of the malaria vector Anopheles gambiae" was retracted in 2015. Reasons: contaminated cell lines or tissues; errors in the data; unreliable results or conclusions.

## Results

### Host choice assay

The attraction of *An. gambiae* and *An. quadriannulatus* laboratory strains to human odor vs cow odor was examined in a dual choice olfactometer. Consistent with the host preference of these species in the field and with recent work on laboratory colonies [40], *An. gambiae* was significantly attracted to human odor (77%, N = 770, p < 0.0001), whereas *An. quadriannulatus* significantly prefers cow odor (67%, N = 330, p = 0.0029). Therefore, the natural host preference of these species is largely preserved in strains kept in laboratory conditions for many generations.

### Gene expression analyses

Three replicate female antennae RNAseq data sets and two replicate maxillary palps RNAseq data sets were obtained for both *An. gambiae* and *An. quadriannulatus.* After quality control screening, 91.0% of antennal reads from *An. gambiae* and 87.0% of antennal reads from *An. quadriannulatus* mapped to the *An. gambiae* reference genome. For palps, 86.8% of the *An. gambiae* reads and 84.3% of the *An. quadriannulatus* reads mapped back to the genome. A higher percentage of total reads obtained for the antennae mapped to a single location in *An. gambiae* vs *An. quadriannulatus* (83.7% vs 78.7%), whereas fewer reads from the palps mapped to only one location for this species (65.6% vs 76.4%). Additionally, the mapping software reported that no *An. quadriannulatus* reads remained unmapped due to mismatches with the reference genome, hence the difference in read mapping is not due to a divergence between the genomes of the two species.

We obtained 58.7 to 79.8 million mapped reads for each of the six antennal samples, for a total of 429.5 million mapped reads. Between 52.3 and 75.0 million mapped reads were obtained for each of the four maxillary palp samples, for a total of 261.9 million. Clustering of the variance-stabilized transformed counts shows that for both antennae and maxillary palp samples there was relatively little variation among biological replicates relative to differences among tissues and species (Additional file 1: Figure S1).

A total of 9,258 and 9,385 annotated genes were detected in the antennae of *An. gambiae* and *An. quadriannulatus* respectively. Of these, 2,593 (28.0%) are significantly higher expressed (q value of < 0.05) in antennae of *An. gambiae* and 2,778 (29.6%) in the antennae of *An. quadriannulatus* (Figure 1A). In the maxillary palps, 9,824 and 9,994 genes are expressed in *An. gambiae* and *An. quadriannulatus,* respectively*.* Of these, 1,243 (12.6%) genes are significantly up-regulated in *An. gambiae* and 1,517 (15.2%) in *An. quadriannulatus* respectively (Figure 1B).

The article "Species-specific chemosensory gene expression in the olfactory organs of the malaria vector Anopheles gambiae" was retracted in 2015. Reasons: contaminated cell lines or tissues; errors in the data; unreliable results or conclusions.

**Figure 1:** **Differential gene expression between** ***An. gambiae*** **and** ***An. quadriannulatus*** **in antennae (A) and maxillary palps (B).** The expression of genes indicated in red is statistically significant (q < 0.05).

A gene ontology analysis (GO) was conducted to recover descriptions of molecular and biological function. For this analysis only significantly enhanced genes that were more than 2-fold expressed were considered. This resulted in 564 antennal genes in *An. gambiae* and 608 antennal genes in *An. quadriannulatus* (Figure 2, Additional file 2: Figure S2). For the maxillary palps, 870 and 787 genes met these criteria in the two respective species (Additional file 3: Figure S3). Of these, 217 genes are shared between the antenna and palps of *An. gambiae,* and 292 of these genes are shared between tissues in *An. quadriannulatus* (Additional file 4: Figure S4). Not surprisingly, some of the gene ontology (GO) terms recovered in the significantly enhanced genes are connected to olfaction (e.g., “odorant binding”) and signal transduction (e.g., “response to stimulus”, “signal transducer activity”). Additionally, we found strong representation of terms connected to enzymatic activity. For example, “transferase activity” represents 7% of the up-regulated genes in the antennae of *An. gambiae* and 5% of those in the maxillary palps of this species (Figure 2, Additional file 3: Figure S3).

**Figure 2:** **GO analysis of 564** ***An. gambiae*** **genes with > 2-fold antennal expression compared to** ***An. quadriannulatus*** **, predicting their involvement in molecular functions (A) and biological processes (B).** Data are presented as level 3 GO categorization. Categories with less than 1% of representation were grouped in “others”.

### Olfactory receptors

Out of the 76 annotated olfactory receptors (*Ors*), 65 were detected above the threshold in the antennae of at least one species (Additional file 5: Table S1). As expected, the co-receptor *Orco* is highly expressed in both *An. gambiae* and *An. quadriannulatus* female antennae (1,429 and 1,756 RPKM, respectively), but is significantly higher in *An. quadriannulatus* (q = 0.025) (Additional file 5: Table S1). Consistent with this observation, the total expression of the specific *Ors* is higher in this species as well (1,738 vs 2,183 RPKM)*,* which is also reflected in the regression slope (1.20) for *Or* expression between species.

A total of 17 *Ors* are expressed at a significantly higher level in *An. gambiae* female antennae (Table 1, Figure 3]. The expression level of *Ors* with significantly enhanced expression in *An. gambiae* ranged from 2.5 to 42.8 RPKM, but *Or36, 45, 66, 69, 70,* 73 and *75* are noteworthy for being both relatively abundant (>12.3 RPKM) and substantially up-regulated (>1.9-fold) in *An. gambiae*. Two expressed *Ors* (*Or8* and *51*) were not expressed in the antennae of *An. quadriannulatus,* but these were among the least abundant *Ors* in *An. gambiae* as well (2.5 and 2.7 RPKM, respectively).

The article "Species-specific chemosensory gene expression in the olfactory organs of the malaria vector Anopheles gambiae" was retracted in 2015. Reasons: contaminated cell lines or tissues; errors in the data; unreliable results or conclusions.

**Table 1:** **Olfactory and gustatory genes that are significantly enhanced in the female antennae of** ***An. gambiae*** **vs** ***An. quadriannulatus***

Gene	***An. gambiae***rpkm	***An. quadriannulatus***rpkm	Fold change	Log2 change	q
*Or8*	2.49	0.65	4.10	1.891	0.000
*Or51*	2.72	0.82	3.54	1.735	0.000
*Or66*	14.09	4.66	3.19	1.640	0.000
*Or69*	29.29	10.54	2.93	1.546	0.000
*Or70*	18.65	6.85	2.87	1.509	0.000
*Or73*	29.01	14.51	2.11	1.065	0.000
*Or65*	2.87	1.43	2.12	1.025	0.000
*Or45*	12.23	6.23	2.05	1.022	0.000
*Or43*	5.52	2.79	2.07	1.019	0.000
*Or28*	2.71	1.39	2.09	1.010	0.000
*Or71*	8.45	4.39	2.04	1.007	0.000
*Or75*	41.79	22.98	1.92	0.934	0.000
*Or36*	21.83	12.10	1.89	0.906	0.000
*Or54*	2.81	1.71	1.73	0.763	0.000
*Or76*	10.02	6.61	1.60	0.675	0.000
*Or22*	15.59	10.33	1.59	0.665	0.000
*Or81*	71.66	61.77	1.22	0.282	0.013
*Ir7s*	2.31	0.04	53.50	4.696	0.000
*Ir75k*	24.50	4.66	5.49	2.433	0.000
*Ir75h.2*	84.23	17.74	4.94	2.283	0.000
*Ir7w*	58.56	16.27	3.81	1.922	0.000
*Ir41n*	56.57	17.75	3.40	1.743	0.000
*Ir93a*	52.93	17.31	3.24	1.687	0.000
*Ir100a*	56.35	18.44	3.24	1.684	0.000
*Ir7u*	7.06	2.29	3.26	1.680	0.000
*Ir7t*	18.64	6.99	2.82	1.482	0.000
*Ir41c*	18.82	7.20	2.77	1.460	0.000
*Ir100i*	4.82	2.13	2.39	1.211	0.000
*Ir7i*	3.38	1.88	1.88	0.901	0.000
*Ir75g*	25.84	14.85	1.84	0.871	0.000
*Ir41t.2*	19.90	13.55	1.56	0.631	0.000
*Ir100h*	4.04	2.81	1.53	0.602	0.000
*Obp10*	2759.9	1222.8	2.36	1.23	0.00
*Obp1*	12041.9	5645.9	2.23	1.15	0.00
*Obp3*	13545.9	7739.3	1.84	0.87	0.00
*Obp7*	18361.3	13074.8	1.47	0.56	0.00
*Obp15*	523.8	336.5	1.63	0.70	0.00
*Obp26*	318.5	127.7	2.65	1.36	0.00
*Obp5*	14868.2	12083.9	1.29	0.37	0.00
*Obp25*	649.0	440.2	1.55	0.63	0.00
*Obp13*	321.7	221.5	1.56	0.62	0.00
*Obp2*	7817.9	7090.3	1.16	0.21	0.00
*Obp56*	2.2	1.2	1.97	0.90	0.00
*Gr52*	7.83	0.40	19.70	4.185	0.000
*Gr51*	3.65	0.55	6.62	2.698	0.000
*Gr49*	2.55	0.44	5.87	2.524	0.000
*Gr48*	2.50	0.68	3.70	1.876	0.000
*Gr24*	4.78	1.75	2.73	1.456	0.000
*Gr50*	1.77	0.69	2.56	1.365	0.000
*Gr23*	4.75	1.91	2.49	1.346	0.000

**Figure 3:** **Regression plot of gene expression between the antennae of** ***An. gambiae*** **and** ***An. quadriannulatus*** **for odorant receptors (A), ionotropic receptors (B), odorant binding proteins (C) and gustatory receptors (D).** Axis represent Ln(RPKM) values. Inset box shows regression line based on non-transformed data. Genes whose expression was significantly different are indicated in black.

The article "Species-specific chemosensory gene expression in the olfactory organs of the malaria vector Anopheles gambiae" was retracted in 2015. Reasons: contaminated cell lines or tissues; errors in the data; unreliable results or conclusions.

In contrast to *An. gambiae,* twenty-eight specific *Ors* are expressed at a significantly higher level in the female antennae of *An. quadriannulatus*. In this species *Or1, 9, 23, 33, 46, 61,* and *63* stand out by being both highly expressed (RPKM >17.3) and substantially enhanced (>2.0-fold). Four *Ors* (*Or18, 20, 30* and *74*) are expressed only in the antennae of *An. quadriannulatus*, although at low levels (1.1 < RPKM < 6.42).

Although no abundant *Ors* are uniquely expressed in the antennae of either species, our analysis identifies a set of *Ors* that show clear species-specific enhancement of their antennal expression. Despite these specific differences, a linear regression analysis shows that overall antennal *Or* expression is highly correlated between the two species with (*R*^*2*^ = 0.937, slope = 1.20, Figure 3A).

Strikingly, the overall expression of *Ors* is much higher in the palps of *An. quadriannulatus* compared to *An. gambiae.* For example, *Orco* is expressed at 187.3 and 700.1 RPKM in *An. gambiae* and *An. quadriannulatus* respectively, and the regression slope for *Or* expression between the two species is 2.84 (Figure 4A). This 2.8 to 3.7-fold enhancement of olfactory receptors expression implies a relatively larger importance of the maxillary palps in the olfaction system of *An. quadriannulatus*.

**Figure 4:** **Regression plot of gene expression between the maxillary palps of** ***An. gambiae*** **and** ***An. quadriannulatus*** **for odorant receptors (A), ionotropic receptors (B), odorant binding proteins (C) and gustatory receptors (D).** Axis represent Ln(RPKM) values. Inset box shows regression line based on non-transformed data. Genes whose expression was significantly different are indicated in black.

That being said, *Ors* are expressed at much lower level in the palps than in the antennae for both *An. gambiae* (slope = 0.105, Figure 5A) and *An. quadriannulatus* (slope = 0.236, Figure 6A). The number of detected *Ors* is also substantially less in the maxillary palps. Only 45 specific *Ors* were detected in the palps of *An. gambiae*, whereas 53 are present in the *An. quadriannulatus* female palps (Additional file 6: Table S2). Interestingly, one olfactory receptor, *Or52,* is unique to the maxillary palps of *An. gambiae*. This gene is among the seven most abundant *Ors* in this species (9.55 RPKM), but did not reach our detection threshold in *An. quadriannulatus* (0.83 RPKM)*.* Furthermore, this gene is all but undetectable in the antennae of either species (0.13 and 0.18 RPKM, Additional file 5: Table S1).

The article "Species-specific chemosensory gene expression in the olfactory organs of the malaria vector Anopheles gambiae" was retracted in 2015. Reasons: contaminated cell lines or tissues; errors in the data; unreliable results or conclusions.

**Figure 5:** **Regression plot of gene expression between the antennae and maxillary palps of** ***An. gambiae*** **and for odorant receptors (A), ionotropic receptors (B), odorant binding proteins (C) and gustatory receptors (D).** Axis represent Ln(RPKM) values. Inset box shows regression line based on non-transformed data. Genes whose expression was significantly different are indicated in black.

**Figure 6:** **Regression plot of gene expression between the antennae and maxillary palps of** ***An. quadriannulatus*** **and for odorant receptors (A), ionotropic receptors (B), odorant binding proteins (C) and gustatory receptors (D).** Axis represent Ln(RPKM) values. Inset box shows regression line based on non-transformed data. Genes whose expression was significantly different are indicated in black.

*Or* expression in the antennae and palps is highly correlated in *An. gambiae* (*R*^*2*^ = 0.80, Figure 5A), but considerably less so in *An. quadriannulatus* (*R*^*2*^ = 0.57, Figure 6A). Of the 17 *Ors* significantly enhanced in *An. gambiae* antennae*,* most are enhanced in the palps of this species compared to *An. quadriannulatus* as well. However, there are two notable exceptions; *Or8,* which shows 3.8-fold up-regulation in the *An. gambiae* antennae, is expressed 4.9-fold higher in the palps of *An. quadriannulatus.* It is also one of most abundant *Ors* in the palps of this latter species. Similarly, *Or28* is significantly 2.0-fold enhanced in *An. gambiae* antennae, but 6.1-fold enhanced in the palps of *An. quadriannulatus* where it is the second most highly expressed specific *Or.*

Not surprisingly, given the 2.8-fold higher overall level of *Or* expression*,* 20 specific *Ors* are significantly enhanced in the palps of *An. quadriannulatus* vs. *An. gambiae.* With the exception of *Or8* and *Or28,* these are also enhanced in the antennae of this species, or are not expressed in either (*Or3* and *5*). Overall, the correlation between *Or* expression in the palps (*R*^*2*^ = 0.80, Figure 4A) of the two species is less than for the antennae (*R*^*2*^ = 0.94, Figure 3A).

### Ionotropic receptors

The total antennal expression of *Irs* is similar between species (1,283 vs 1,232 RPKM in *An. gambiae* and *An. quadriannulatus* respectively), with a regression slope of 1.07 (Figure 3B). Of the 44 annotated *Irs,* 29 are expressed in the female antennae of *An. gambiae* and 32 are expressed in *An. quadriannulatus* (Additional file 5: Table S1). *Ir25a,* one of the co-receptors, is by far the most highly expressed *Ir* in both species. However, both species also express *Ir76b* at very high levels. This gene has been considered a putative co-receptor [26], but which was more recently proposed to encode a Na^+^ leak channel which in *Drosophila* also plays a role in salt detection [41]. A total of 15 *Irs* are significantly up-regulated in *An. gambiae* antennae, with nine (*Ir75h.2, 7t, 7w, 41c, 41n, 75g, 75k, 93a,* and *100a*) standing out by being both considerably enhanced (>1.8-fold), as well as among the more abundant *Irs* (Figure 3A, Additional file 5: Table S1). Twelve *Irs* are significantly enhanced in the female antennae of *An. quadriannulatus.* Only two specific ionotropic receptors*, Ir75d* and *75h.1*, are considerably up-regulated (>1.9-fold) and abundant (>19.5 RPKM) in this species. Similarly to *Or* expression, *Ir* expression is highly correlated between species (*R*^*2*^ = 0.79, Figure 3B).

The article "Species-specific chemosensory gene expression in the olfactory organs of the malaria vector Anopheles gambiae" was retracted in 2015. Reasons: contaminated cell lines or tissues; errors in the data; unreliable results or conclusions.

The total *Ir* expression is much lower in the palps than the antennae (slope = 0.115 for *An. gambiae,* Figure 5B, and 0.384 for *An. quadriannulatus*, Figure 6B)*,* but like the *Ors* is much higher in *An. quadriannulatus* (regression slope = 3.7, Figure 4B). Twenty-four *Irs* are expressed in the palps of *An. gambiae*, of which only *Ir101* is significantly 3.1-fold enhanced in this species, but it is expressed at very low levels in the palps (and antennae) of both species (Table 2, Additional file 6: Table S2). None of the 15 significantly enhanced *Irs* in *An. gambiae* antennae are significantly enhanced in its palps. The expression of eight *Irs* is significantly enhanced in the palps of *An. quadriannulatus.* Six of these are also significantly enhanced in the antennae of this species. *Ir* expression in the palps is highly correlated between the two species (*R*^*2*^ = 0.89, Figure 4B), as well as between the antennae and palps of the two species, with *R*^*2*^ = 0.92 for *An. gambiae* and *R*^*2*^ = 0.98 *An. quadriannulatus* (Figures 5B and 6B) (See Table 3).

**Table 2:** **Olfactory and gustatory genes that are significantly enhanced in the female**

Gene	***An. gambiae***rpkm	***An. quadriannulatus***rpkm	Fold change	Log2 change	q
*Or52*	9.55	0.83	14.92	3.255	0.000
*Ir101*	1.01	0.41	3.10	1.459	0.003
*Obp26*	337.15	202.39	2.10	1.046	0.000
*Obp56*	13.03	7.30	2.23	1.108	0.001
*Gr49*	24.20	0.35	68.36	5.591	0.000
*Gr51*	15.20	0.63	23.96	4.535	0.000
*Gr52*	13.88	0.65	21.25	4.421	0.000
*Gr48*	18.60	0.83	22.29	4.240	0.000
*Gr50*	11.05	0.84	13.16	3.663	0.000
*Gr25*	1.72	0.64	2.66	1.368	0.004

Maxillary palps of *An. gambiae* vs *An. quadriannulatus.*

**Table 3:** **Summary of olfaction/gustation genes whose expression is significantly different between** ***An. gambiae*** **and** ***An. quadriannulatus*** **, and those who are also > 2-fold expressed**

Gene Family	Tissue	***An. gambiae***		***An. quadriannulatus***	
		Significant	> 2-fold	Significant	> 2-fold
Olfactory Receptors	Antennae	17	11	27	13
	Maxillary Palps	1	1	21	21
Ionotropic Receptors	Antennae	15	11	12	5
	Maxillary Palps	1	1	8	8
Odorant Binding Proteins	Antennae	11	2	5	2
	Maxillary Palps	2	2	14	13
Gustatory Receptors	Antennae	7	7	7	6
	Maxillary Palps	6	6	9	9

The article "Species-specific chemosensory gene expression in the olfactory organs of the malaria vector Anopheles gambiae" was retracted in 2015. Reasons: contaminated cell lines or tissues; errors in the data; unreliable results or conclusions.

### Odorant binding proteins

As expected based on OBP function, *Obp* expression in the antennae is considerably higher than that of the *Ors* and *Irs* (as much as 51,541.1 RPKM in *An. gambiae* and 61,872.7 RPKM in *An. quadriannulatu*s, Figures 3C and 4C). In fact, *Obp48* is by far the most highly expressed gene in the antennae of both species, and nine of the top 15 most highly expressed genes are *Obps* (Additional file 5: Table S1)*.* That being said, only 27 and 29 of the 57 putative *Obps* were detected in *An. gambiae* and *An. quadriannulatus* female antennae*.*

The overall level of antennal *Obp* expression is similar in *An. gambiae* and *An. quadriannulatus* (183,218 vs 172,629 RPKM, slope = 1.08, Figure 3C). Expression of eleven *Obps* is significantly enhanced in *An. gambiae* female antennae, and three abundant odorant binding proteins, *Obp1, 3* and 10 are more than 1.8-fold enhanced in this species (Table 1). The expression of five *Obps* was significantly higher in *An. quadriannulatus,* but of the three that were considerably up-regulated (>1.9-fold), only *Obp19* was expressed at any appreciable level (464.8 RPKM). Similarly to *Or* and *Ir* expression, antennal *Obp* expression was highly correlated between species (*R*^*2*^ = 0.95, Figure 3C).

Also consistent with *Or* and *Ir* expression, the *Obp* abundance in the palps is considerably lower than in the antennae (slope = 0.133 for *An. gambiae* and 0.411 for *An. quadriannulatus,* Figures 5C and 6C). Again similar to *Or* and *Ir* expression, the overall *Obp* expression is several folds higher in the palps of *An. quadriannulatus* as compared to *An. gambiae* (slope = 3.39, Figure 4C). Furthermore, *Obp48,* the most abundant gene in the antennae of both species, ranks 8th in *An. gambiae* maxillary palps in abundance, whereas it is also the most highly expressed of all genes in *An. quadriannulatus.*

One relatively abundant odorant binding protein, *Obp26* (337.2 RPKM)*,* is expressed at significantly higher levels in *An. gambiae* palps (2.1-fold), and is also significantly up-regulated in the antennae of *An. gambiae*. Not surprisingly given the 3.4-fold higher level of overall *Obp* expression in *An. quadriannulatus* palps, 14 *Obps* are significantly enhanced in this species, including *Obp48* (Figure 4C, Additional file 6: Table S2). However, the correlation between *Obp* expression in the palps of the two species is high (*R*^*2*^ = 0.95, Figure 4C), and there is also a strong correlation between *Obp* expression in the antennae and palps for both species (*R*^*2*^ = 0.90 for *An. gambiae* and *R*^*2*^ = 0.88 for *An. quadrianulatus,* Figures 5C and 6C).

The article "Species-specific chemosensory gene expression in the olfactory organs of the malaria vector Anopheles gambiae" was retracted in 2015. Reasons: contaminated cell lines or tissues; errors in the data; unreliable results or conclusions.

### Gustatory receptors

The gustatory receptors (*AgGrs*) are expressed at very low levels in the antennae of both species, with total RPKM values of 57 and 71 in *An. gambiae* and *An. quadriannulatus* respectively (Figures 3D and 4D, Additional file 5: Table S1). None-the-less, the expression of seven *AgGrs* is significantly enhanced in *An. gambiae,* and the same number is significantly up-regulated in *An. quadriannulatus.* Interestingly, five *AgGrs* that are significantly enhanced in *An. gambiae* (*AgGr48-52*) are not expressed in *An. quadriannulatus,* although the expression of these genes in *An. gambiae* is low as well, ranging from 1.8 to 7.8 RPKM. To compare, ranking these with the *Ors* in level of abundance would place *AgGr52* in 44^th^ position. Two *AgGrs, AgGr1* and *AgGr26,* stand out in the *An. quadriannulatus* antennal dataset. They are relatively abundant in this species (8.7 and 21.3 RPKM) and significantly up-regulated (>2.6-fold). In contrast to the olfaction gene families, little correlation exists between *AgGr* expression in the antennae of the two species (*R*^*2*^ = 0.01, Figure 3D).

Only 18 out of 60 annotated *AgGrs* are expressed in the palps of *An. gambiae,* and 15 are expressed in *An. quadriannulatus* palps (Figure 4D, Additional file 6: Table S2). The three *AgGrs* responsible for CO_2_ detection in mosquito palps (*AgGr 22, 23 and 24*) are by far the most highly expressed *AgGrs* in *An. quadriannulatus.* Interestingly, the expression level of these CO_2_ receptor genes is between 5.1 and 6.1-fold higher in this species*,* but is on par with the expression of other *AgGrs*, such as *AgGr48* and 49, in *An. gambiae.* Overall the regression slope between the two species for the palps is 3.03 (Figure 4D), indicating a much higher expression in *An. quadriannulatus,* but this is entirely due to the CO_2_ receptors.

Probably the most striking result from the palp data set is a set of species-specific *AgGrs* in *An. gambiae.* The five up-regulated gustatory receptors from the *An. gambiae* antennae (*AgGr48-52*) are in fact highly abundant in the palps of this species (11.1 < RPKM < 24.2, Table 2). Interestingly, they are all but absent from the palps of *An. quadriannulatus* (<0.84 RPKM)*.*

The article "Species-specific chemosensory gene expression in the olfactory organs of the malaria vector Anopheles gambiae" was retracted in 2015. Reasons: contaminated cell lines or tissues; errors in the data; unreliable results or conclusions.

Similarly, four *AgGrs* (15, 17, 21, and 26) are abundant and up-regulated in *An. quadriannulatus* palps (9.5 < RPKM < 24.7, > 4.9-fold). These genes are all at very low levels in *An. gambiae* palps, with *AgGr26* being unique to *An. quadriannulatus.* Interestingly, this gene is also expressed at high levels in the antennae of *An. quadriannulatus* (21.3 RPKM).

## Discussion

Because of *An. gambiae’*s odor-mediated host seeking behavior [1], it is expected that its preference for human hosts has a strong genetic basis in its olfactory system. This system is primarily housed in the antennae, but the maxillary palps are also involved [14]. In this study a comparison of the olfactory organ transcriptomes of the anthropophilic *An. gambiae* and its zoophilic sibling species *An. quadriannulatus* identified species-specific patterns of olfaction gene expression. Even though the expression profiles of olfaction genes are highly correlated between species, clear differences were observed which identify olfaction genes that may play an important role in differential host preference.

The olfactory system of *Anopheles* mosquitoes plays a role in at least two other aspects of their biology; finding a sugar source, most often nectar, and identifying oviposition sites. No data is available on how often or from what source *An. quadriannulatus* females obtain sugar meals. However, *An. gambiae* starts ignoring honey volatiles five days after emergence and responds almost exclusively to human odor at that point [42]. Our experience in the laboratory indicates that *An. quadriannulatus* also switches to host seeking around this time. The larval ecology of both species appears to be similar, with both breeding in shallow, open, sunlit fresh water pools [43, 44], and in any case oviposition-site searching does not commence until 48 hours post-blood feeding. Therefore, although we cannot rule out that the differences in olfaction gene expression between the two species are due to biological differences other than host-seeking, there is no data to suggest that such differences are substantial. In addition, the use of 6-day old females in our study optimizes our ability to detect differences in olfaction gene expression that are related to host-seeking [45].

In the antennal transcriptome, seven *Ors* (*Or36, 45, 66, 69, 70, 73, 75*) and nine *Irs* (*Ir75h.2, 7t, 7w, 41c, 41n, 75g, 75k, 93a, 100a*) stand out by being among the more highly expressed receptor genes, while also being considerably up-regulated in *An. gambiae* (1.8 to 4.7-fold)*.* We speculate that the enhanced expression of some of these genes in *An. gambiae* contributes to an increased sensitivity to human odor. Divergence in olfaction gene expression associated with host specialization has been observed between closely related *Drosophila* species that feed on different host plants. Antennal expression of *Or*s differed markedly between the generalists *D. melanogaster, D. simulans*, and their specialist sister-species *D. sechellia*, and as many as 53% of the *Or*s were differentially expressed between species pairs [32].

The article "Species-specific chemosensory gene expression in the olfactory organs of the malaria vector Anopheles gambiae" was retracted in 2015. Reasons: contaminated cell lines or tissues; errors in the data; unreliable results or conclusions.

Previous studies have examined the response of 56 *AgOrs* to a wide range of odorants [24, 25]. These included 11 of the 17 *Ors* enhanced in *An. gambiae* in the present study. Only four receptors showed a positive response to any of the tested odorants. The exposure of *Or75* to eight human volatiles led to a small to moderate increase in the firing rate of the neuron [24]. *Or36* has a very narrow tuning curve and responded strongly to only two of the tested odorants, however neither of which are of human origin [25]. *Or65* responded mildly to one human odorant (4 methylphenol), as well as to several other chemicals [24]. Finally, *Or8* on the other hand responded strongly to two known human odorants, 1-octen-3-ol and 1-hepten-3-ol [24, 25]. However, for many of these human volatiles it is not known if they are unique to humans. For example 1-octen-3-ol is exhaled by bovids as well, and is a common compound produced by mushrooms [46]. Finally, it should be kept in mind that 346 volatiles have been identified in human sweat [7], and only a small subset of these volatiles were tested on these *Ors.*

Expression differences in *Obps* may also play a role in the human host preference of *An. gambiae*. Several highly expressed *Obps* (*1*, *3, 10*) are enhanced (1.8 to 2.4-fold) in the antennae of *An. gambiae*, whereas no abundant *Obps* are substantially higher expressed in *An. quadriannulatus.* The presence of specific odorant-binding proteins is well-known to impact behavior in *Drosophila.* Flies carrying LUSH, a mutant OBP, are defective in detecting an aggregation pheromone [47], and *Obp57d* and *Obp57e* are involved in differences in oviposition behavior between *Drosophila* species [48].

Importantly, our data shed new light on the role of the maxillary palps in odor detection in these species. Lu et al. [14] concluded that a relatively small repertoire of *Ors* is responsible for olfaction coding in the maxillary palps, although it was found that in *Culex quinquefasciatus* the maxillary palps are broad spectrum odorant detectors [49]. A previous analysis of the transcriptome of *An. gambiae* maxillary palps indicated the expression of relatively small *Or* repertoire [20], with only four *Ors* expressed at >1 RPKM. Those data contrast with our results, in which 49 *Ors* were detected in the palps of this species. Although it is not clear at what level the expression of receptors is biologically relevant, 19 of these *Ors* are expressed at > 4 RPKM, suggesting the palps may be able to detect a suite of odors. Possible reasons for these contrasting results between the two studies may be that we conducted our dissections during the early dark cycle, and included replicates, which is recommended for obtaining reliable RNAseq data [50].

The article "Species-specific chemosensory gene expression in the olfactory organs of the malaria vector Anopheles gambiae" was retracted in 2015. Reasons: contaminated cell lines or tissues; errors in the data; unreliable results or conclusions.

Another interesting feature of our data is the several fold higher overall expression of the three olfaction gene families in the maxillary palps of *An. quadriannulatus* compared to *An. gambiae.* Clearly, the maxillary palps of *An. quadriannulatus* are considerably more important component of this species’ olfactory olfaction system than is the case for *An. gambiae.*

While no *An. gambiae* specific olfaction genes were identified in the antennae, an analysis of the maxillary palp transcriptome revealed several *An. gambiae* specific chemosensory genes. *Or52,* the seventh most abundant *Or* in the *An. gambiae* palps, is not expressed in *An. quadriannulatus.* Interestingly, this gene is also absent from the antennae of *An. gambiae*. This indicates that this maxillary palp receptor could play a species-specific role in *An. gambiae’s* biology, and thus may possibly be involved in human host preference. Unfortunately, this *Or* was not including in the odorant affinity studies discussed above [24, 25].

Additionally, the expression pattern of several *AgGrs* indicates that they play a species-specific role in olfaction. *AgGr48-52* are specific to *An. gambiae,* and these five *AgGrs* are expressed at relatively high levels in the maxillary palps*,* indicating a functional role of the receptors encoded by these genes. With the exception of *AgGr22-24,* which together encode the heteromeric CO_2_ receptor [14, 51], gustatory receptors are generally considered to be primarily involved in gustation. However, the fact that *AgGr48-52* are expressed in both the antennae and maxillary palps of *An. gambiae* suggests a role in olfaction for these genes. These genes are located in tandem on the chromosome 2R and each pair is separated by only 46 to 326 bp. Therefore, the expression of these genes is likely controlled by the same regulatory elements. Additionally, *AgGr26* is specific to *An. quadriannulatus.* It is expressed at high levels only in the maxillary palps and the antennae of this species, suggesting a species-specific role. Therefore, these gustatory receptors may play a significant role in the behavioral differentiation between *An. gambiae* and *An. quadriannulatus*.

The article "Species-specific chemosensory gene expression in the olfactory organs of the malaria vector Anopheles gambiae" was retracted in 2015. Reasons: contaminated cell lines or tissues; errors in the data; unreliable results or conclusions.

The several fold higher expression of olfaction genes in the palps of *An. quadriannulatus* dominates the comparison between the palps of the two species. Nevertheless, *Obp26* and *Obp56* are more than 2-fold enhanced in the maxillary palps of *An. gambiae.* Interestingly, both are enhanced in the antennae of this species as well, although *Obp56* is expressed at very low levels in this organ.

Several other noteworthy observations result from these data. The expression of *Orco* and the *Ors* is 18% to 26% higher in the antennae of *An. quadriannulatus.* Although the antennal sensilla of *An. quadriannulatus* were found to outnumber those of *An. gambiae,* their density is actually similar in both species [52], indicating that this difference is not explained by differences in the antennal morphology. Furthermore, the overall level of *Ir* and *Obp* expression is actually slightly higher in *An. gambiae* antennae. This implies that the overall sensitivity to the odorants detected by *Ors* is higher in *An. quadriannulatus* antennae.

The expression of the CO_2_ receptor genes *AgGr22-24* in the maxillary palps of both species differs markedly. These genes are expressed between 5.1-6.1 fold higher in *An. quadriannulatus*, which greatly exceeds the overall higher level of expression of olfaction genes in the palps of this species. By itself, CO_2_ is a poor attractant to *An. gambiae.* It does activate and guide it towards a human odor source, but at this point other semiochemicals become important [53]. In contrast, CO_2_ is highly attractive to *An. quadriannulatus,* which has a more catholic host preference [38]. Our data suggest that the lesser attraction of *An. gambiae* to CO_2_ is accompanied by a lower sensitivity to CO_2_. It has been suggested that anthropophilic mosquitoes primarily use CO_2_ to detect hosts as a long distance cue [54]. Given the smaller amount of CO_2_ produced by a human vs. the preferred host of *An. quadriannulatus*; a bovid, and the relatively low expression level of the CO_2_ receptor genes in *An. gambiae*, this species either relies little on CO_2_ for its long range attraction, or is incapable of detecting hosts from the same distances as *An. quadriannulatus.*

Although the *An. quadriannulatus* strain examined in this study showed a preference for bovine hosts, this species did not distinguish between human and cow sweat in an olfactometer in a previous study [4]. Furthermore, when offered a choice of a human or equal sized calf, it blood fed equally on both [3]. This suggests that *An. quadriannulatus* has a wider host preference and is more of a generalist than *An. gambiae.* This is consistent with its much higher level of expression of the CO_2_ receptor genes. However, the large number of olfaction genes with enhanced expression in *An. quadriannulatus* indicates that it, like *An. gambiae,* likely responds to a complex blend during host seeking, similar to *An. gambiae* [12, 55].

The article "Species-specific chemosensory gene expression in the olfactory organs of the malaria vector Anopheles gambiae" was retracted in 2015. Reasons: contaminated cell lines or tissues; errors in the data; unreliable results or conclusions.

Rinker et al. [36] recently compared the daytime transcriptomes of the antennae of *An. gambiae* and *An. quadriannulatus.* Their results correspond roughly with ours. A linear regression analyses of the day-time olfaction gene expression with the early dark phase reported here, resulted in R^2^ values of 0.74-0.78 for the three olfaction gene families in *An. gambiae,* and 0.76-0.91 in *An. quadriannulatus.* That being said, a few notable exceptions were observed. For example, the expression differences for *Or66*, *73* and *Obp26* was much less pronounced during the daytime. For a few genes, *e.g. Ir75k, 7t* and *75g* the expression pattern was even reversed*.* Similarly, several olfaction genes showed differential expression during the day-time, but not during dark cycle (e.g. *Obp2* and *13*). The expression of *Orco* and a variety female antennae *Obps* in female *Anopheles gambiae* fluctuates throughout the circadian cycle. Expression of these olfaction genes was generally found to be highest during the early stage of the dark phase, and therefore seems to be correlated with the female’s host seeking activity [37]. However, a comparison between light and dark cycle transcriptomes, suggests that the expression pattern of olfaction genes do not all follow the same diel expression cycle.

Ionotropic receptors have been divided into “antennal” and “divergent” IRs depending on whether they are expressed in the antennae of *Drosophila* [16]. It was suggested that this distinction held across a wide range of insects and that divergent IRs play a predominant role in gustation rather than olfaction. Additionally, it was found that antennal IRs tend to be more conserved than the divergent IRs. However, this classification has limited relevance to the expression pattern observed in the antennae of *An. gambiae*. Of the expressed *Irs*, 17 were classified as antennal, and 14 as divergent IRs, although of the 14 *Irs* not expressed in the antennae, 12 are divergent IRs.

## Conclusion

Our data identifies potential human host preference genes in the malaria vector *An. gambiae,* but also provides new insight into the importance of the maxillary palps in the olfactory system. The palps are where the most dramatic difference in chemosensory gene expression is observed between the anthropophilic *An. gambiae* and the zoophilic *An. quadriannulatus,* with several highly expressed receptor genes that are specific to either species. Finally, the expression patterns of several *AgGrs* strongly suggest a species-specific role for them in the olfaction system of *An. gambiae.*

The article "Species-specific chemosensory gene expression in the olfactory organs of the malaria vector Anopheles gambiae" was retracted in 2015. Reasons: contaminated cell lines or tissues; errors in the data; unreliable results or conclusions.

### Ethics statement

Colonies of Anopheles mosquitoes were kept following the Arthropod Containment Guidelines established by The American Committee of Medical Entomology of the American Society of Tropical Medicine and Hygiene. The behavioral experiments were conducted in the Laboratory of Entomology at Wageningen University in the Netherlands. Approval to obtain an odor sample from a cow was obtained from the Animal Use Committee of Wageningen University.

## Methods

### Mosquito rearing

Laboratory strains of *An. gambiae* M form (GASUA), recently proposed to be named *An. coluzzii* [56], and originally collected in Suakoko, Liberia, as well as *An. quadriannulatus* (SANQUA) established from female mosquitoes collected in Sangwe, Zimbabwe were reared in the insectaries at Wageningen University, The Netherlands (host choice experiment) and Texas A&M University, College Station, TX, USA (RNAseq analyses). Rearing conditions were 25°C, 75-85% relative humidity and a light:dark photoperiod of 12 hours. Female mosquitoes were blood fed on defibrinated rabbit blood using a membrane feeding system. Larvae were maintained at densities of approx. 150 per 2 L container and fed finely ground fish food (Tetramin, Melle, Germany). Pupae were collected and placed into cages at densities of two cups of 150 pupae per cage.

For mosquitoes used in RNAseq analyses, cages were checked daily for newly emerged mosquitoes. To ensure mosquitoes were the same age, pupae that did not eclose were transferred to new cages. Male and females mosquitoes were kept together in a cage and fed a 5-10% sucrose solution for six days until tissue dissections. Hence, females were given an opportunity to mate, but not to blood-feed. We checked the insemination rate in 50 *An. gambiae* females at day 6 and found it to be high (82%).

### Dual odor-choice assay

A total of 750 female *An. gambiae* and 330 *An. quadriannulatus* females were tested to determine the odor preference of the two species in laboratory conditions. Mosquitoes were put at a density of 75–80 in release cages for use in a dual-choice olfactometer [57] the night before experiments, and provided with a wet cotton ball for hydration. Human and cow odor traps were prepared on the morning of the experiments. Human odor was derived from the socks worn by volunteers for 24 hours, and cow odor was derived from a panty hose tied around the leg of a cow for 24 hours. Odor sources were switched between the left and right port of the olfactometer between runs. A single, centrally placed CO_2_ plume was used as activator. Conditions during the experiments were as follows: temperature = 26-28°C, humidity 55-75% inside olfactometer, 80% in front of port holes, air-speed 018–0.22 ms^−1^, and released [CO_2_] = 4.5%. Mosquitoes were released into the olfactometer during the dark-cycle for 15 min. under semi-dark conditions. Mosquitoes remaining in the wind tunnel after the experiment were disposed of.

The article "Species-specific chemosensory gene expression in the olfactory organs of the malaria vector Anopheles gambiae" was retracted in 2015. Reasons: contaminated cell lines or tissues; errors in the data; unreliable results or conclusions.

### Molecular methods

Female mosquitoes were killed shortly after the start of the dark cycle by placing them at −20°C. This is when anophelines begin their host searching activity and when *Orco* expression in *An. gambiae* peaks during the circadian rhythm [37]. The antennae and maxillary palps were removed from frozen mosquitoes placed on dry ice and were stored in RNAlater^*®*^ (Ambion). Between 600 to 800 6-day old females were dissected for each replicate and three replicates per species were included for a total of six samples per species. Samples were stored at 4°C for 24 hours, before RNAlater was removed and stored at −80°C until RNA extraction.

Total RNA was isolated from each sample using miRNeasy (Qiagen) columns according to the protocol supplied by Qiagen. RNA quantity was initially verified using a Qubit fluorometer (Life Technologies). Next, RNA was further quantified using a NanoDrop spectrophotometer (Thermo Scientific) and the quality assessed using RNA Pico LabChip analysis on an Agilent BioAnalyzer 2100 (Agilent Technologies) by the Agrilife Genomics Center at Texas A&M University.

mRNA was isolated from 1 μg of total RNA and cDNA libraries were prepared using an Illumina TruSeq RNA Library kit (Illumina). Each single-end library contained two/three replicates that had been given a unique tag using barcode sequences supplied by the library kit. Each library was sequenced on a single lane of an Illumina flow cell and using 50 cycles on an Illumina HiSeq 2000. Preparation and sequencing of libraries were both performed by the University at Buffalo Next-Generation Sequencing and Expression Analysis Core Facility. Approximately 50–70 million reads with an average read of 51 base pairs were generated for each replicate sample and used for further analysis.

### RNA sequencing analyses

Read quality was assessed using FastQC (ver 0.10.0) and processed using NGS QC toolkit [58] with at least 80% of the reads had Phred > 30 (raw reads Phred quality score 0–40). Reads were trimmed and then filtered by length, discarding reads < 40 bp. Sequencing reads were mapped to the reference *An. gambiae* genome (AgamP3; December 2013) using the software package STAR [59]. Alignments were discarded if they had more than two mismatches. Read counts were conducted with HTSeq-count (ver 0.5.4) (http://www.huber.embl.de/users/anders/HTSeq/doc/count.html). Only reads that aligned to a unique location in the genome were used to calculate the expression levels. Sequence data was obtained for three replicates of the antennae for each species, and for three replicates for the palps. One palp replicate for each species provided poor quality data, and these were therefore discarded from further analyses. Tests for differential expression in the female antennae or palps from *An. gambiae* versus *An. quadriannulatus* were performed in the R package DESeq2 [60]. Size factors for each dataset were calculated to normalize library sizes across replicates, and overall means and variances were determined using a negative binomial distribution model. Genes were considered to be differentially expressed if q < 0.05 after correcting for multiple testing. Genes were considered not expressed if RPKM <1.

The article "Species-specific chemosensory gene expression in the olfactory organs of the malaria vector Anopheles gambiae" was retracted in 2015. Reasons: contaminated cell lines or tissues; errors in the data; unreliable results or conclusions.

To compare the tissue and species effect on the overall gene expression, we computed the correlation coefficient (R^2^) and slope from a linear regression between *An. gambiae* versus *An. quadriannulatus* data sets, as well as between maxillary palps and antennae. Scripts used to run RNAseq analyses are presented in Additional file 7. Reads for *Obp6* and *Obp29* mapped to multiple locations in the genome, therefore expression data for these two genes are unreliable, and not considered in this analysis.

### Gene ontology analysis

Genes that met the following criteria: q < 0.05, FoldChange > 2, RPKM > 1 at least in one sample, between antenna and maxillary palps of *An. gambiae* versus *An. quadriannulatus* were used for gene ontology (GO) analyses. GO Annotation was performed using Blast2GO [61]. The gene sequences were retrieved from Ensembl Genomes release 22 via Biomart (http://metazoa.ensembl.org/index.html). GO annotation was used for assessment of the genes differentially expressed in each sample. GO annotation associates analyzed transcripts with terms from hierarchical vocabularies describing, e.g., molecular function or biological process.

### Availability of supporting data

All fastq files containing the raw data were deposited at the NCBI Sequence Read Archive. [http://www.ncbi.nlm.nih.gov/sra?term=SRP050131]. The full gene expression data are available in “Additional file 5” (antennae) and “Additional file 6” (maxillary palps).

## Electronic supplementary material

Additional file 1: Figure S1: PCA plot showing the antennal and maxillary palps data sets of *An. gambiae* and *An. quadriannulatus* in the 2D plane spanned by their first two principal components. (PDF 41 KB)

Additional file 2: Figure S2: GO analysis of 608 *An. quadriannulatus* genes with >2-fold antennal expression compared to *An. gambiae*, predicting their involvement in molecular functions **(A)** and biological processes **(B)**. Data are presented as level 3 GO categorization. Categories with less than 1% of representation were grouped in “others”. (PDF 128 KB)

Additional file 3: Figure S3: GO analysis of 870 *An. gambiae* genes with >2-fold maxillary palp expression compared to *An. quadriannulatus*, predicting their involvement in molecular functions **(A)** and biological processes **(B)**, and of 787 *An. quadriannulatus* genes with >2-fold maxillary palp expression compared to *An. gambiae*, predicting their involvement in molecular functions **(C)** and biological processes **(D)**. (PDF 247 KB)

Additional file 4: Figure S4: Venn diagram showing the overlap in the number of genes significantly and more than 2-fold higher expressed in the tissues of either species. (PDF 79 KB)

Additional file 5: Table S1: Gene expression data for all genes in the antennae of *An. gambiae* and *An. quadriannulatus.* (XLSX 2 MB)

Additional file 6: Table S2: Gene expression data for all genes in the maxillary palps of *An. gambiae* and *An. quadriannulatus.* (XLSX 2 MB)

Additional file 7: **Scripts used to run RNAseq analyses.** (DOCX 110 KB)
